# Aesthetic Characteristics of Dance Based on Few-Shot Learning and Neural Networks

**DOI:** 10.1155/2022/4740234

**Published:** 2022-06-29

**Authors:** Dixin Qu

**Affiliations:** Shandong University (Weihai), Weihai 264200, China

## Abstract

Dance is constantly discovering truth, goodness, and beauty in human social life, spreading truth, goodness, and beauty, and fully expressing the artistic pursuit of dance beauty. It shapes different dance images, expresses the aesthetic consciousness and feelings of dance, and resonates with the audience to meet their aesthetic needs through various forms of movement. Because the RBF neural network model is good at approximating functions, many researchers have begun to use the RBNN approximation model for engineering design. Due to the limited dance data available for research, this paper uses radial basis function neural network model to study the aesthetic characteristics of dance in the context of few-shot learning. When the time index reaches 50, the average ratio of the L-MBP algorithm is 33.4 percent, 32.5 percent for the RBNN algorithm, and 46.3 percent for this method. As can be seen, this method has the highest ratio of the three algorithms, giving it a distinct advantage in terms of dance aesthetics. As a result, this paper establishes a neural network model, trains and simulates the network model, studies and analyzes the influence of changes in influencing factors on the aesthetic characteristics of dance, and provides a new idea for the prediction of the aesthetic characteristics of dance and a reference for optimizing the design of the aesthetic system of dance using the prediction ability of radial basis function neural networks.

## 1. Introduction

Dance existed as a form of culture long before it was considered aesthetically pleasing. The evolution of cultural dance to aesthetic dance has become a historical necessity as time passes, productivity improves, and class emerges. The emergence of dance with aesthetic significance not only makes dance an art in the strict sense but also gradually forms a dance art discipline, and then produces a new discipline—dance aesthetics. Dance art incisively and vividly seeks out truth, goodness, and beauty in human social life; spreads truth, goodness, and beauty; and embodies the artistic pursuit of dance beauty. It shapes various dance images, expresses the aesthetic consciousness and aesthetic emotion of dance through various action forms, resonates with the audience, and meets their aesthetic needs through various action forms [1]. Don't you know that when you dance with beautiful eyes, a slim waist, and graceful hands and feet, your beautiful posture of expressing feelings and ideas is like flowing sculptures, shocking, and fascinating enough to arouse the viewer's resonance and reverie? Is n't this a one-of-a-kind dance language? The artistic effect of “silence is better than sound at this time” can often be obtained by the visual beauty of the image without saying anything. Dance, in contrast to Chinese national folk dance, transcends cultural boundaries. The inheritance and promotion of Chinese traditional culture, Chinese national temperament, and Chinese classical spirit are primarily reflected in its aesthetic characteristics. Dance beauty is a pleasurable psychological state in which people use their vision, hearing, and other senses to perceive, comprehend, and taste the dance image and spiritual needs. Only those with the ability to appreciate things can generate “aesthetic feelings” in the realm of sound. Aesthetics must also have a certain amount of imagination. Dance, in addition to vertical absorption, horizontally absorbs some characteristics of other art forms, and dance itself is constantly changing and developing, resulting in new developments in the dance inheritance, but it never changes, and the inheritance of Chinese national temperament and dance spirit is always the main vein of dance [2]. The more the life experience is, particularly life experience related to specific works, the more conducive to art appreciation one has. As far as dance appreciation is concerned, the appreciator should also know something about the characteristics, types, styles, and different styles of dance art, which is conducive to the in-depth feeling and comprehension of dance works. Being able to correctly discover, recognize, and evaluate beauty is the basic aesthetic ability to learn dance art. Therefore, in dance teaching, the study of dance aesthetic characteristics is closely related to improving students' aesthetic ability.

Because the RBF neural network model [3] is good at approximating functions, many researchers have begun to use the RBNN approximation model for engineering design. The radial basis function neural network is a feedforward neural network with only one hidden layer that can realize the hidden layer's nonlinear mapping and the output layer's linear mapping. The action function of the radial basis function neural network's hidden layer node generates a local response to the input signal. The hidden layer node produces a large output when the input signal is close to the basis function's central range. According to the RBF neural network model, the RBF neural network's training algorithm is investigated, and the K-means clustering algorithm is used to determine the hidden layer node center, hidden layer node width, and output weight of the network, as well as the network model framework [4]. The impact of the number of hidden layer nodes and distribution coefficient on the accuracy of the RBF neural network model is investigated using an empirical formula and a comparative test method, and the two parameters are finally determined to complete the RBF neural network model's establishment.

The dance focuses on “quietness,” “harmony” is the most important, the coordination between breathing and body is emphasized, the harmony and unity between every detail is emphasized, and a kind of harmony and coordination is emphasized in the dance movements. This kind of adduction and harmony of dance comes from the Chinese character, characteristics of “harmony is the most important thing” and “the beauty of neutralization,” and it is a highlight of the Chinese nation's aesthetic psychology. Its round, curved, twisted, and inclined posture and circular track of movements can well reflect the Chinese philosophical spirit of repeated cycles and constant renewal [5]. Therefore, with the help of the prediction ability of radial basis function neural network, this paper establishes a neural network model, trains and simulates the network model, studies and analyzes the influence of the changes of influencing factors on the aesthetic characteristics of dance, and provides a new idea for the prediction of the aesthetic characteristics of dance and a reference for optimizing the design of the aesthetic system of dance. Under the radial basis function neural network model, the aesthetic characteristics of dance are mainly embodied in original ecology, where original ecology is relative to performance and folk, and folk is relative to the former court [6]. Folk of dance refers to the folk customs and nationality reflected from dance movements and dance images, and the nationality of dance refers to the common national style, temperament, and spirit reflected from dance movements and dance images. Folk is the foundation of nationality, and nationality is folk. The innovations in this paper are as follows:

1. This paper constructs the model diagram of radial basis function neural network. RBF neural network model reflects the nonlinear evolution relationship of the overall structure through repeated learning of sample data, so as to predict the unknown data. Therefore, the training sample data are very important for the fitting accuracy and generalization ability of neural network.
2. The aesthetic characteristics of dance are tested and analyzed. When the time index reaches 50, the average proportion of L-MBP algorithm is 33.4%, the average proportion of RBNN algorithm is 32.5%, and the average proportion of this method is 46.3%. It can be seen that the proportion of this method in the three algorithms is the highest, so it plays a greater advantage in the aesthetic characteristics of dance.

The overall structure of this paper consists of five parts. The first section introduces the background and significance of dance aesthetic characteristics, and then introduces the main work of this paper. The second section mainly introduces the research status of dance aesthetic characteristics at home and abroad. The third section introduces the radial basis function neural network model. The fourth section introduces the aesthetic characteristics of dance and the analysis of the experimental part. The fifth chapter is the summary of the full text.

## 2. Research Status of Aesthetic Characteristics of Dance at Home and Abroad

So put forward that when people's inner feelings reach the point where language and words cannot express them, they cannot help dancing and expressing their inner feelings. This kind of progressive emotional expression from low to high just reflects that dance, as a “silent art,” has surpassed such vocal languages as poetry and music, and has become the highest level of emotional expression, reflecting the strong lyrical aesthetic characteristics of dance art [7]. Habron and Merwe put forward that dance images are mainly figures, animal and plant images, or morphological objects created by dancers through their movements. Image is an important aesthetic feature of dance [8]. Christmas in dance teaching, capturing vivid dance images, is the premise and foundation of dance learning [9]. K. Skjoldager-Nielsen and D. Skjoldager-Nielsen put forward that this dance feature is also the inheritance of ancient Chinese dance. In ancient Chinese dance, people like to get close to the Earth or the site, and the dancers are mainly focused on gaining momentum. Generally, they rarely raise their feet, but move their feet slowly along the intended geometric figure, which is in favor of the ever-changing movements of arms and hands [10]. Lustig and Tan put forward that in dance teaching, it is important for students to understand and master the aesthetic characteristics and types of dance lyricism to improve their aesthetic ability [11]. Anderson put forward that accumulating rich life experience and artistic practice experience, going deep into the folk to carry out art gathering activities, being good at discovering and digging beauty from life, and absorbing rich nutrition from the “root” of dance art are important methods to capture dance images and enhance aesthetic ability, so as to better serve the shaping of dance images [12]. A. Wang and C. Wang proposed that many original ecological folk dances are formed within the same nation due to different branches, geographical distribution, economic status, and cultural development. These seemingly different original ecological folk dances have the nationality of the same nation and reflect the same aesthetic psychology and aesthetic habits [13]. Schuh proposed that the shape of dance occupies space and the melody of music occupies time. The audience's appreciation of dance must first be accepted through vision. Visibility has become a feature of dance aesthetics [14]. Jürgens puts forward that the aesthetic characteristics of ethnic minority dance are mainly embodied in performance, nationality, and folk. Both academic folk dance and ethnic minority dance have the characteristics of performance, nationality, and folk. Their dance movements are derived from the dance movements of original folk dance, which have been processed, refined, integrated, and transcended [15]. Adewale proposed that the aesthetic feature of dance is lyricism. Dance is good at lyricism and bad at narration. Only when poetry, song, and music are not enough to express feelings can we “dance with hands and dance with feet” [16].

Based on the above analysis, this paper puts forward a radial basis function neural network model to study the aesthetic characteristics of dance and then uses the improved optimal stop training method to control the training of these two parameters so that the established prediction model can obtain better generalization ability. Under the radial basis function neural network model, human body movements can only be developed into dance language with dance artistic attributes after people's artistic processing and creation in accordance with the regularity and purpose of dance aesthetic features, and can only become a tool for shaping dance images and a means of expressing dance so that the beauty of dance works can be planed and embodied on this basis. The dance features in the aesthetic features of dance reflect the psychological characteristics of outward development, the belief in God, and the commonness of Western traditional culture. Of course, this psychological feature of outward development is inseparable from the geographical environment in the west. Under the aesthetic characteristics of dance of radial basis function neural network model, the enthusiastic and unrestrained mental state of the actors and the rhythm of their feet with a sense of the times make the audience feel the pulse and rhythm of modern life psychologically, and bring people's thoughts to a brand-new realm, so as to arouse people's inner pursuit of beauty and inspire people's strong love for life, work, and study. The expression in the radial neural network model is the soul of form through facial expressions and body expressions. As the saying goes, “superb” means this. Therefore, in the performance, students should follow the principle of “taking the shape with the spirit,” “expressing the spirit with the shape,” and “having both the form and the spirit,” as well as the artistic law of “taking the lead with the spirit before the body moves, and arriving with the spirit when the shape fails.”

## 3. Radial Basis Function Neural Network Model

### 3.1. Principle and Algorithm of Radial Basis Function Neural Network

Radial basis function neural network is a feedforward neural network based on interpolation algorithm, which can approximate any nonlinear function with any accuracy [17]. Compared with BP network, the excitation function of RBF neural network is radial symmetric function, which only responds to the input signal locally, so it avoids the problem of long training time and easy to fall into local minimum of BP network. RBF neural network model reflects the nonlinear evolution relationship of the overall structure through repeated learning of sample data, so as to predict the unknown data. Therefore, the training sample data are very important for the fitting accuracy and generalization ability of neural network. When selecting sample data, we pay attention to the following three points:

① The sample data should be widely distributed, covering the whole structure of the problem and fully reflecting the potential law.
② The sample data should be distributed evenly to avoid the phenomenon of too dense local data.
③ Remove the impossible data, so as to prevent it from generating data noise and affecting the convergence of the network.

In the work of multilayer perceptron neural network, the function coincidence is imminent, which is defined by the nested function set of the weighted sum of input and threshold value, and the weight matrix is calculated through recursive iteration, and the output is calculated. Different from other feedforward neural networks such as MLP, the working principle of RBF neural network function fitting is to map the input directly to the high-dimensional space, and then carry out a single linear weighting and output in the output layer, so that the supervision and training time of weights are greatly reduced [18, 19]. In radial basis function neural network, the number of nodes in the input layer is consistent with the input dimension of the learning sample, while the number of nodes in the output layer is consistent with the output dimension of the actual problem. Therefore, once the learning sample is determined, the number of nodes in the input layer and the number of nodes in the output layer are determined at the same time [20]. The input layer node only transmits the input signal to the hidden layer. After the nonlinear transformation of the hidden layer node, the output is generated by the linear function of the output layer node. The neural network model consists of three layers, and its structure is shown in Figure 1.

The first layer is the input layer, which consists of signal source nodes. The number of input nodes is the dimension of the input sample. Assuming that there are *N* input samples, each input sample is a *I* dimension column vector, that is, *X*=(*x*_1_, *x*_2_,…,*x*_1_)^*T*^, and each element of the sample column vector is the node of the input layer. The second layer is the hidden layer, and the number of neurons in the hidden layer varies with the application to be solved. The activation function of each hidden node adopts radial basis function. Radial basis function is a kind of non-negative nonlinear function, which is symmetrical about the center point and attenuates radially, and it has local response function. The third layer is the output layer, which responds to the output of the hidden layer. Assuming that the number of nodes in the output layer is *K*, this layer maps the hidden layer space to the output layer. Because of the special properties of radial basis function, it has the selective response ability to input variables, which makes RBF network to have the local tuning ability. We take the hidden layer action function as Gaussian function, and the hidden layer output is

(1) $$\begin{array}{c} R_{i}\left(x\right)=\exp\left(-\frac{{\left\|X-C_{i}\right\|}^{2}}{2\sigma_{i}^{2}}\right),i=1,2,\ldots ,h, \end{array}$$

where *h* is the number of neurons in the hidden layer; *X*=(*X*_1_, *X*_2_,…, *X*_*k*_) is the *k* dimensional input vector; *C*_*i*_ and *σ*_*i*_ are the center vector and width of the *i*th radial basis function in the hidden layer; ‖∘‖ is the 2 norm, representing the Euler distance between *X* and *C*_*i*_; and *R*_*i*_(*X*) is the output of the *i* radial basis function. The output of the whole RBF neural network is

(2) $$\begin{array}{c} y_{j}=\sum_{i=1}^{h}w_{ji}R_{j}\left(X\right),j=1,2,\ldots ,c_{i}=1,2,\ldots h, \end{array}$$

where *y*_*j*_ is the output of *j* neuron in the output layer, and *w*_*ji*_ is the connection weight between *i* neuron in the hidden layer and *j* neuron in the output layer.

Let *MN* be the number of hidden nodes, *CN* be the number of original clusters of samples, and *β* be the redundancy coefficient of hidden nodes. Its value can be determined according to the network learning situation, and it is generally acceptable as 0 < *β* < 0.5. The number of hidden nodes of radial neural network can be determined by formula.

(3) $$\begin{array}{c} MN=CN+\beta \circ CN. \end{array}$$

In order to speed up the training of RBF neural network, it is necessary to initialize the center and width of hidden layer RBF appropriately. The center of hidden layer neurons is intuitively taken as the class mean value. The selection of width takes into account the dispersion of samples within the class and the distance between classes. If the dispersion of samples within the class is large or the distance between classes is large, the width of radial basis function shall be larger; otherwise, it shall be smaller, and its value shall be determined according to the formula.

(4) $$\begin{array}{c} \sigma_{i}=d_{dj}-d_{j}^{\text{inner}}=m_{i}n\left\|C_{i}-C_{j}\right\|-\sqrt{\frac{1}{Y_{i}|{\sum_{x\in Y}{\left\|X-C_{i}\right\|}^{2}}_{i}}}, \end{array}$$

where *d*_*ij*_ is the distance between class center *C*_*i*_ and *C*_*j*_, *m* is the number of classes, *d*_*j*_^inner^ is the dispersion degree within classes, *X* is the sample point within class *Y*_*i*_, and |*Y*_*i*_| is the total number of samples in class *Y*_*i*_.

The basic idea of this algorithm is that the response of hidden layer nodes in radial basis function neural network to input depends on the distance between the input vector and the center of hidden layer nodes. The smaller the distance between the input vector and the center, the greater the response of hidden layer nodes. Therefore, the process of determining the hidden layer nodes is the process of clustering the input samples according to the distance between samples. The input vectors with small distance from each other belong to the same category, and the clustering center is the center of the hidden layer nodes. Different network structures and weight training algorithms lead to different characteristics and application functions of the network. At the early stage of neural network development, the network structure was simple, with only input layer and output layer, and its application was single. The emergence of multilayer neural networks [21–23] is the inevitable result of the development of neural networks [24]. Besides the input layer and the output layer, the middle layer of the multilayer neural network is called the hidden layer, which can be one or more layers. The radial basis neural network is composed of radial base layer and linear output layer, and the first layer is radial base layer, which is composed of radial basis neurons. The second layer is a linear output layer composed of linear neurons. The structure diagram of radial neural network model is shown in Figure 2.

In Figure 2, *R* is the dimension of the input vector, *S*^1^ is the number of neurons in the radial base layer, *S*^2^ is the number of neurons in the linear output layer, and IW_1,1_ represents the IW_1,1_ row element of the weight matrix *i*. ‖dist‖ is the Euclidean distance between the input vector *P* and the weight matrix IW_1,1_, so the output vector consists of *S*_1_ elements, which are the distance between the input vector *P* and the vector IW_1,1_ composed of the row vectors of the input weight matrix.

The expression of radial neuron transfer function is shown in formula.

(5) $$\begin{array}{c} a=\text{radbas}\left(n\right)=\exp\left(-n^{2}\right). \end{array}$$

The input *n* of the transfer function is the product of the weighted input ‖*w* − *P*‖ and the offset *b*, *w* is the weight vector of the radial basis function neuron, and *p* is the input vector. The distribution coefficient SPREAD of radial basis function is defined as 0.8326/*b*, so the output *a* of radial basis function neurons can be expressed as follows:

(6) $$\begin{array}{c} a=\text{radbas}\left\{0.8326\times \frac{w-p}{\text{SPREAD}}\right\}. \end{array}$$

When ‖*w* − *p*‖ is equal to SPREAD, *n* is 0.8326, and the output *a* of neurons is exactly 0.5. When ‖*w* − *p*‖ is greater than SPREAD, neurons will produce less than 0.5 output; when ‖*w* − *p*‖ is less than SPREAD, neurons will produce an output higher than 0.5. The above is the mathematical significance of radial basis function distribution coefficient.

In order to facilitate processing, we use root mean square error (RMSE) to describe the average level of *Q* cross-validation errors

(7) $$\begin{array}{c} \text{RMSE}=\sqrt{\frac{1}{Q}\sum_{\text{i}=1}^{Q}cve_{i}^{2}}. \end{array}$$

To sum up, when the training sample is given, the root mean square error (RMSE) is actually a function with the distribution coefficient SPREAD as the independent variable.

*v*_*i*_ represents the *i* element of vector *v*, and *M*_*i*_ represents the *i* row of matrix *M*; then, there is the following relationship:

(8) $$\begin{array}{c} n_{i}^{1}=\left\|{\left({\text{IW}}_{i}^{1,1}\right)}^{T}-p\right\|b_{i}^{1};i=1,\ldots ,S^{1}, \end{array}$$

(9) $$\begin{array}{c} a_{i}^{1}=\text{rabdas}\left(n_{i}^{1}\right);i=1,\ldots ,S^{1}, \end{array}$$

(10) $$\begin{array}{c} y_{i}=a_{i}^{2}={\text{IW}}_{i}^{2,1};a^{1}+b_{i}^{2};i=1,\ldots ,S^{2}. \end{array}$$

It can be seen from the above formula that for a given input vector *p*, the output vector FF of RBF neural network can be completely determined according to IW^1,1^, *b*^1^, LW^2,1^, *b*^2^, and *y*.

The RBF neural network maps the input to the high-dimensional space by calculating the functional of the distance function between the input and the point in the hidden layer; that is, it completes the mapping by activating the function. The activation function is the basis function, which is radially symmetrical about a central point of the dimensional space. The activation degree of the input at the hidden layer neuron has a strong correlation with its distance from the middle, so this hidden layer node has “local characteristics.”

### 3.2. Characteristics of Dance Beauty

Dance art is a comprehensive art that includes lyricism, movement, and image. To better understand dance, we must not only improve our aesthetic ability in dance but also our aesthetic ability in related arts. This will allow us to better appreciate the formal beauty of dance. Dance's history reveals that it coexists with human history and keeps pace with human social development, which is why it is so popular. As a result, its purpose is socially significant. Many countries now include dance in their school curricula. Dance classes have been offered in some university elective courses, which are very popular with young students, despite China's late start. It demonstrates that people's perceptions of dance's social function have been greatly enhanced. Nowadays, high speed and efficiency are valued in modern civilized life. The information society and the electronic world are icons of the industrial era, and they have had a significant influence on the original dance form. People prefer strong, powerful, heroic, and confident dancing when this psychological factor is in control. They perform a series of complex dance steps in a short amount of time, including rapid and colorful rotation, and rapid twisting. At the same time, people's aesthetic feelings about dance works are inextricably linked to the beauty of dance; however, people's subjective feelings must be grounded in the objectively existing beauty of dance, which must possess the basic characteristics of originality, craftsmanship, and comprehensiveness. This kind of originality is the result of a lot of sweat and hard work, and it is attained through a lot of hard study and exploration, even after a lot of failures. All of this reflects a spiritual beauty, and it is admirable. The created dance image can give people an aesthetic feeling, and this unique skill is beyond the reach of ordinary people.

In a dance work, first of all, it should have aesthetic characteristics such as originality, skill, and comprehensiveness, so as to give people a feeling of dance beauty, be loved by people, and be called excellent dance works. “Form and spirit, spirit and rhyme” is to analyze the aesthetic characteristics of dance movements through the research category of dance aesthetics, and it shows that the improvement of dance aesthetic ability plays an important role in teaching. Dance expresses thoughts through the moving human body, and the human body movements are linked by emotional logic. Like poetry and music, it has the structural method of literary thoughts. The structure of the article is words, words, sentences, paragraphs, and chapters, and the structure of dance is dancing, dancing, dancing, dancing, and dancing. Although in the long history, poetry, music, and dance have gradually taken an independent development path, and their respective artistic characteristics have been relatively highlighted, their internal relationship, that is, comprehensiveness, has never been interrupted or independent, and they have always maintained a state of “you and me” or “you and me.” For dance, this phenomenon is more obvious and prominent.

As the external form of dance beauty, after having the artistic attribute of dance, the dance image must also go through the comprehensive development of dance aesthetic creation, that is, the integration of dance, music, poetry, and other different arts, so as to better understand the aesthetic attribute of dance, and finally complete the aesthetic of dance. Dance is embodied by a unique rhythm of “force.” The movement of dance is the movement of “Qi.” It is the rhythm of “force” of human body's “Qi” sensing the “Qi” of the universe. All dances should use the internal “Qi” to show the external “force.” With the help of the research on the aesthetic characteristics of dance, this paper demonstrates the important role of dance aesthetic ability in dance teaching, which can provide some enlightenment to the theory and practice of dance teaching. There is a lack of exploration and innovation in artistic conception and artistic expression; that is, there is no originality; instead, the old routine is adopted in a light and familiar manner or in a conventional manner, and the performance is the theme and content that we have seen and understood for a long time. There will be no new ideas for people, and bringing beauty to people is impossible. As a result, dance must possess unique aesthetic characteristics. Dance serves as a vehicle for moral and emotional education. Real, kind, and beautiful feelings, wishes, and ideals of choreographers and dancers are reflected in the pleasing dance image. It has a subtle positive effect, cultivating people's temperament, evoking noble sentiment, inspiring emotion, inspiring fighting spirit, and so on. Because dance is a form of art in which human body movements are the primary means of expression, it is unavoidable that the means of expression of dance become more artistry as the scope of dance performance subjects and the depth of the theme content expands. The colorful life content and rich characters' inner world can only be fully displayed through a high level of artistry. These characteristics are often integrated and penetrated into each other in an excellent dance work, but they are sometimes hidden and sometimes prominent. However, a close examination reveals that these qualities are present in excellent works as well and that they are interdependent or inseparable.

## 4. Simulation and Results

### 4.1. Determination of the Number of Hidden Layer Nodes

In order to establish an ideal dance aesthetic feature model, the commonly used method of gradually increasing the number of hidden layer nodes is adopted to adjust the neural network, and 30, 70, and 120 hidden layer nodes are selected for experiments, respectively, and then, the mean square error between each output variable and the real value is calculated. Tables 1–3 show the mean variance of the output values of the three networks.

From Tables 1to 3, it can be seen that the fitting accuracy of training data is higher and higher with the increase in hidden layer nodes. When the number of hidden layer nodes is the same as the number of training samples, the fitting error of the network to the training set reaches 0. But at this time, the prediction accuracy of the three dance aesthetic feature test sets is not high. However, because the proportion of dance aesthetic feature training samples in the total data is not large, and its absolute accuracy is not low, the interval of the number of hidden layer nodes can be preliminarily determined.

### 4.2. Analysis of Aesthetic Characteristics of Dance

In this experiment, L-MBP algorithm, RBNN algorithm, and this method are used to compare the aesthetic characteristics of dance, and the calculation results of RBNN approximate model are attached in Figure 3. The initial weights of FNN are randomly generated, and the set initial weights directly affect the final training results. The experimental results are shown in Figure 3.

As can be seen from Figure 3, when the conditions other than the initial weight under the aesthetic characteristics of dance are the same, the values of FNN approximate model based on L-MBP algorithm vary greatly; by contrast, when the training sample of dance aesthetic characteristics is given, the quality of RBNN approximate model is only related to the value of distribution coefficient. Once the value of spread is determined, the RBNN approximate model and its values will be completely determined. The RBF neural network model predicts the aesthetic characteristics of dance; that is, the principal component score coefficient is used to calculate the principal component value, and the data of dance aesthetic characteristics are normalized; finally, L-MBP algorithm, RBNN algorithm, and this method are used to establish the RBF neural network of dance aesthetic features in the mapping relationship, which constitutes the proportion of PCA-RBF network. The experimental results are shown in Figure 4.

As can be seen from Figure 4, when the time index reaches 50, the average proportion of L-MBP algorithm is 33.4%, RBNN algorithm is 32.5%, and the average proportion of this method is 46.3%. It can be seen that this method accounts for the highest proportion of the three algorithms, so it plays a greater advantage in the aesthetic characteristics of dance. In order to verify the advantages of radial basis function neural network over other networks, this paper constructs PCA-BP network and uses machine learning, decision tree algorithm, and this method to repredict the aesthetic characteristics of dance. Similarly, 2∼20 groups of data are used as training samples, and 22∼26 groups of data are used to evaluate and test the model. The test simulation results of soft sensor model are shown in Figure 5.

As can be seen from Figure 5, when the time index reaches 60, the average ratio of machine learning algorithm is 44.3%, that of decision tree algorithm is 49.5%, and that of this method is 57.8%. Similarly, the change of this method in the training of dance aesthetic feature errors among the three algorithms is the highest, which proves the feasibility and accuracy of this method. In the experiment, we use the proposed EDIW-PSO algorithm, LDIW-PSO algorithm, NDIW-PSO algorithm, and GLBESTIW-PSO algorithm to optimize the RBF neural network, train the training samples, and obtain the fitness function curves of the four optimization algorithms. When the fitness function reaches the minimum value, the optimal parameter value of neural network obtained by algorithm optimization is shown in the table. The fitness function curves of the four optimization algorithms are shown in Figure 6.

As can be seen from Figure 6, among the four methods, the PSO algorithm, which is an exponential declining inertia weight strategy, has a faster convergence rate, the smallest fitness function value, and the smallest training error of the neural network. The formal beauty of dance art is relatively independent, and formal beauty is one of the common forms of common beauty, which is most likely to cause a common sense of beauty, and the popularity of dance works is also likely to cause people's common sense of beauty. Because of the existence of common aesthetic feeling, good works can transcend national and national boundaries and reflect people's common interests, life ideals, and psychological needs. In this experiment, the changes of dance aesthetic feature fitness function fitting two-dimensional nonlinear function of four models are compared experimentally. EDIW-PSO-GRBF model, NDIW-PSO-ADABOOST GRBF model, LDIW-PSO-ADABOOST GRBF model, and radial basis function neural network model in this paper are used for experiments, respectively. The experimental results are shown in Figure 7.

As can be seen from Figure 7, the radial basis function neural network model in this paper has the fastest convergence speed, and the global optimal solution searched is better than the other four models, with smaller training error. The subjectivity embodied in aesthetic judgment created aesthetic comprehension's subjectivity. Aesthetic comprehension's subjectivity, as a form of rationality, is based on objectivity, but at the same time, it is latent and fuzzy.

## 5. Conclusions

The purpose of the rhythm of movements in dance works is to investigate the rhythm of dance by drawing inspiration from natural phenomena such as river, lake, and sea fluctuations, as well as the flashing of stars in the universe and the swaying of weeping willows by the lake. As a result, we must be adept at recognizing and learning the beauty and inner spirit of rhythm. Based on the RBF neural network model, this paper investigates the aesthetic characteristics of dance. When the time index reaches 50, the average proportion of L-MBP algorithm is 33.4 percent, 32.5 percent for RBNN algorithm, and 46.3 percent for this method. As can be seen, this method has the highest proportion in the three algorithms, so it has a greater advantage in the aesthetic characteristics of dance. The more difficult it will be, the higher the RBF neural network model's skill in dance performance. This is not something that ordinary people can do, which just goes to show how unique dance is in terms of innovation and creativity. With the ever-changing nature of life, dance art will change, develop, and improve, and will play a role in the construction of both material and spiritual civilizations. The simulation of surgery in the radial basis function neural network model can make people happy. On the contrary, the form of simulation content is changing and even deepening with the advancement of society and human civilization. The mode of production, lifestyle, and ideology is changing, much like China's transition from an agricultural to an industrial society, and the dance form and content of the aesthetic characteristics of dance are bound to change as well.

## Figures and Tables

**Figure 1:** Radial basis function neural network model.

**Figure 2:** Structure diagram of radial basis function neural network.

**Figure 3:** Comparison results of approximate models of dance aesthetic characteristics.

**Figure 4:** Error curves of dance aesthetic characteristics under different algorithms.

**Figure 5:** Training curve of dance aesthetic characteristic error under different algorithms.

**Figure 6:** Fitness function curve.

**Figure 7:** Fitness change of dance aesthetic characteristics of four models fitting two-dimensional nonlinear function.

**Table 1:** Mean square error of 30 hidden layer nodes.

30	Test 1	Test 2	Test 3	Train
*L*	4.0276	4.3147	6.582	2.9947
*A*	5.051	4.4913	5.4983	3.2176
*B*	5.6398	5.7176	7.8707	3.3521

**Table 2:** Mean square error of 70 hidden layer nodes.

70	Test 1	Test 2	Test 3	Train
*L*	2.6595	1.9798	2.5888	0.5702
*A*	3.0583	2.7625	3.1556	0.97
*B*	3.5221	2.9441	4.1052	1.0325

**Table 3:** Mean square error of 120 hidden layer nodes.

120	Test 1	Test 2	Test 3	Train
*L*	0.9653	1.0663	1.225	0.1925
*A*	1.2467	1.1262	1.3702	0.2345
*B*	1.3062	1.3823	1.5531	0.2244

## Data Availability

The data used to support the findings of this study are available from the author upon request.
